# An improved beluga whale optimizer—Derived Adaptive multi-channel DeepLabv3+ for semantic segmentation of aerial images

This article has been retracted.

**DOI:** 10.1371/journal.pone.0290624

**Published:** 2023-10-30

**Authors:** Anilkumar P., Venugopal P.

**Affiliations:** School of Electronics Engineering, Vellore Institute of Technology, Vellore, India; Shandong Agricultural University, CHINA

## Abstract

Semantic segmentation process over Remote Sensing images has been regarded as hot research work. Even though the Remote Sensing images provide many essential features, the sampled images are inconsistent in size. Even if a similar network can segment Remote Sensing images to some extents, segmentation accuracy needs to be improved. General neural networks are used to improve categorization accuracy, but they also caused significant losses to target scale and spatial features, and the traditional common features fusion techniques can only resolve some of the issues. A segmentation network has been designed to resolve the above-mentioned issues as well. With the motive of addressing the difficulties in the existing semantic segmentation techniques for aerial images, the adoption of deep learning techniques is utilized. This model has adopted a new Adaptive Multichannel Deeplabv3+ (AMC-Deeplabv3+) with the help of a new meta-heuristic algorithm called Improved Beluga whale optimization (IBWO). Here, the hyperparameters of Multichannel deeplabv3+ are optimized by the IBWO algorithm. The proposed model significantly enhances the performance of the overall system by measuring the accuracy and dice coefficient. The proposed model attains improved accuracies of 98.65% & 98.72% for dataset 1 and 2 respectively and also achieves the dice coefficient of 98.73% & 98.85% respectively with a computation time of 113.0123 seconds. The evolutional outcomes of the proposed model show significantly better than the state of the art techniques like CNN, MUnet and DFCNN models.

## 1. Introduction

Image segmentation is a fundamental issue in computer vision and other image processing applications. Because of its widespread use in a variety of applications, image segmentation has become quite difficult over the years. In recent times, along with the enhancement of the Remote Sensing methodology, the number of Remote Sensing images also become large as well as the resolution has also become higher. Remote Sensing images acquire a lot of useful details, hence there are several features in the applications of Remote Sensing images that have included semantic segmentation, target detection, person detection, Road surface changes, scene categorization and so on. The applications of Remote Sensing images are shown significantly utilized for illegal building extraction, urban planning, and road extraction [1–3]. In this field, there is a requirement for high-quality segmentation. Even though there are various Remote Sensing image segmentation techniques, still there is a need for enhanced segmentation and detection of insulator in aerial images with diverse background inference [4]. Semantic segmentation is defined as the pixel-level categorization technique that makes every pixel in the image to a specific kind of object label.

The semantic segmentation task on Remote Sensing images has faced several difficulties [5]. In the initial stage, the Remote Sensing images have huge information, but the number of data in every sample is not similar as well as the samples over various scenes are diverse which has put forward the higher requirement of segmentation technique [6]. Secondly, when the Remote Sensing images are attained vertically from a high altitude, few samples may occlude and overlap like in the occlusion of trees on vehicles which has resulted in feature differences in vehicle extraction [7]. Thirdly, the similar group of the sample has also diverse characteristics and details like the top color of the building and different color trees in the forest which brings difficulty to the segmentation [8]. Fourth, considering the different angles of the sun, there are numerous shadows in the images that are defined as the noise in the images [9]. Hence, several researchers have paid attention to the segmentation of Remote Sensing images.

Deep CNN has determined the learning ability of feature representation on computer vision. In the case of semantic segmentation, the Fully Convolutional Neural Network (FCN) has shown predominant enhancements when assimilated over other hand-crafted features [10]. As inspired by FCN, a variety of structures and techniques have been recommended to enhance the semantic segmentation process to next level like encoder-decoder architecture using SegNet, DeepLabv2 and spatial pyramid pooling structure on the PSPNet and DeepLabv3+ for semantic segmentation of UAV remote sensing images based on edge feature fusing and multilevel upsampling. Being diverse from the multimedia images, the higher resolution aerial images generally cover a larger area as well as include complex scenes that have brought limitations to the semantic segmentation tasks [11]. In another case, the high-resolution aerial images also contain rich geographical details like Digital Surface Model (DSM). The research work has also recommended that the DSM has the ability to enhance the categorization outcomes [12]. The conventional techniques have been divided into three categories. The image fusion technique has combined DSM, and the near Infrared, Red, and Green (IRRG) spectrum is taken as the input of the network. It has introduced relevant aspects in the training period because it does not show the relation among heterogeneous details. Fusion technique aspects dependent on the parallel branch network has utilized two CNNs in order to process the multispectral data and Lidar point cloud data separately. Moreover, the performance of this technique is dependent on intermediate outcomes as well as the model training. By using this training approach, the detection of the global optimal solution is difficult.

In addition to being used in remote sensing, semantic segmentation is a widely-researched area of computer vision that is also used in many other applications, including face recognition, autonomous driving, medical and biological imaging, retail services, and autonomous vehicles. In medical and biological imaging, there are many trends like in digital image processing of isolated microalgae by incorporating classification algorithm[13]. Reliable image classification by machine learning and deep learning technologies like artificial neural networks, support vector machines, and convolutional neural networks are used to identify different types of microalgae [14]. Regression and artificial neural network analysis of Red-Green-Blue picture components are used to estimate chlorophyll concentration and Cultivation of Chlorella vulgaris on dairy waste in microalgae. The best methods for predicting chlorophyll content were regression and artificial neural networks. When the factors were taken into consideration, artificial neural networks produced excellent results comparable to regression [15–17]. Deep learning techniques have achieved considerable success in the last ten years, particularly in the field of computer vision, and have since established themselves as a go-to tool for several tasks including object identification, artificial intelligence, scene recognition for automation, etc. The fact that these techniques work directly from raw photos as opposed to needing the extraction of characteristics from the images is one of their fundamental advances.

The major objectives of the proposed work are as follows:

- To recommend the new Semantic Segmentation of Aerial Image model with the aid of IBWO and AMC-Deeplabv3+ techniques for attaining betterment in the regularization process over a series of strong baselines over other models.
- To develop the IBWO algorithm with the help of the BWO algorithm for optimizing the parameter in the AMC-Deeplabv3+ as well as useful for Semantic Segmentation of Aerial Images.
- To design the AMC-Deeplabv3+ technique for effectively segmenting the aerial images, where the parameters like epochs as well as the learning rate in the deeplabv3 model for enhancing the working activity of the model by using the IBWO algorithm.
- To provide the maximum dice coefficient as well as accuracy values to make the Semantic Segmentation of Aerial Images effective over other conventional models by using different performance metrics.

The following sections of the segmentation of the aerial images model are detailed as follows. The existing work related to the segmentation of the aerial images model is provided in section 2. Dataset model and system architecture are in section 3. Implementing an improved beluga whale optimizer for optimizing parameters in deep learning segmentation is in section 4. A novel adaptive multichannel deeplabv3+ for effective segmentation of aerial images is in section 5. The attained results for the outcomes of the semantic segmentation model are in section 6. The semantic segmentation conclusion is in section 7.

## 2. Literature survey

### 2.1 Related works

In 2018, Volpi and Tuia [18] suggested a novel technique in order to learn all forms of pieces of evidence in the semantic class likelihoods and semantic boundaries across shallow-to-deep visual features and classes through the multi-task CNN architecture. They have concatenated the bottom-up details along with the top-down spatial regularization, which has been encoded with the aid of a conditional random field model that has optimized the label space across the segments along with the constraints related to spatial, data-dependent pair-wise as well as the structural relationship among the regions. The outcomes have shown that such strategies have given betterment in the process of regularization over the series of strong baselines reflecting ultra-modern methods. The recommended techniques have offered principled as well as flexible frameworks in order to include various sources of structural and visual information on permitting different degrees of spatial regularizations accounting for priors about the expected model.

In 2019, Luo et al. [19] recommended a new Deep Fully Convolutional Network (DFCN) along with the Channel Attention Mechanism (CAM-DFCN) for attaining high-resolution aerial image semantic segmentation. This model has followed the architectural mode of encoder-decoder. The CAM has been addressed to manually weigh the channel of the feature map to perform the feature selection techniques. Moreover, the CAM has followed the concatenated feature maps on every level in order to select more discriminative features for categorization. On the other hand, the encoders, two similar deep residual networks (DRN) have been split into several levels. Further, the feature map concatenation has been made over every level. The CAM has utilized further weighing the semantic details as well as the spatial position details in the adjacent-level concatenated features maps for more effective predictions. The estimation of the recommended CAM-DFCN has been performed by utilizing datasets. Then, the experimental outcomes have also been attained with considerable improvement.

In 2019, Cao et al. [20] recommended the Digital Surface Models (DSMs) details as the complementary features to enhance the semantic segmentation outcomes. In the end, the recommended simple as well as light weighted DSM fusion (DSMF) structure modules were designed. when assimilated over the conventional feature extraction techniques, the recommended DSMF module has simple as well as be easily applied to other networks. Additionally, the proposed model has four fusion phases that have been dependent on the DSMF module to explore the optimal feature fusion techniques, as well as the DSMFNets, which have been modelled in accordance with the corresponding strategies. The estimation of this model has shown promising outcomes in terms of accuracy.

In 2020, Liu et al. [21] have recommended the network structure as well as designed the Atrous Spatial Pyramid Pooling (ASPP) technique for retrieving the multi-scale features from the various training phases of the target. The inception blocks were utilized in order to strengthen the width of the network that has the potential to attain more abstract features without losing the depth of the network. Moreover, the backbone network has utilized the semantic fusions in the context; hence it has retained more spatial features, as well as the effective decoder network, was developed. At the end, the designed model was evaluated over given dataset. The outcomes have also shown that the network has higher performance.

In 2021, Gupta et al. [22] have recommended techniques that used the segmentation neural network to detect the impacted areas as well as access roads in post-disaster scenarios. The efficiency of the pre-training along with the ImageNet-for the task of aerial images segmentation has been demonstrated as well as its performance of popular segmentation models has been assimilated. The investigational outcomes have shown that the pre-training on the ImageNet has usually enhanced the segmentation process for numerous models. The open data attained from the Open Street Map (OSM) has been utilized for the training phase, forgoing the need for time-consuming manual annotations. This method has also utilized the graph theory in order to update the road network data available from OSM as well as to identify the changes caused by natural disasters. Extensive investigation of the data has also shown the efficiency of the recommended model.

In 2021, Abdollahi et al. [23] recommended the Generative Adversarial Network (GAN) dependent deep learning techniques for road segmentation through high-resolution aerial images. The generative part of the recommended GAN techniques has utilized the modified UNet model (MUNet) to attain the high-resolution segmentation map of the road network. In integration with the simple pre-processing comprising edge-preserving filtering, the recommended techniques have provided enhancement on the road network segmentation assimilated along with the prior techniques. On assimilating over other techniques, the recommended techniques have demonstrated the recommended GAN framework outperforming the CNN dependent and it is specifically effective in preserving edge details.

In 2021, Girisha et al. [24] have recommended the CNN mode through incorporating the temporal details to enhance the effectiveness of the video semantic segmentation process. Here, the improved encoder-decoder dependent CNN model (UVid-Net) has been recommended for the purpose of Unmanned Aerial Vehicle (UAV) video semantic segmentation. The encoder in the recommended model has integrated the temporal details for performing temporary labelling process. The decoder has been improved by implementing the feature-refiner module that was used in the relevant localization techniques of the labels. The recommended UVid-Net architecture for UAV video semantic segmentation has been estimated over extended datasets. The working performances of metric mean IoU were attained that was greater over other algorithms. Moreover, the recommended model has produced promising outcomes even for the pre-trained models.

In 2022, Pei et al. [25] have suggested a novel multi-scale aware-relation Network (MANet) to tackle the problem of intense variations of scenes and object scales in remote sensing. They investigated discriminative and diverse multi-scale representations inspired by the process of human perception of multi-scale (MS) information. They have proposed an inter-class and intra-class region refinement (IIRR) method for discriminative Multi-Scale representations to reduce feature redundancy caused by fusion. IIRR guides Multi-Scale fine-grained features using refinement maps with intra-class and inter-class scale variation. Then, to increase the diversity of Multi-Scale feature representations, propose multi-scale collaborative learning (MCL). At the end, based on the dispersion of multilevel network predictions the segmentation results were rectified.

In 2022, Diao et al. [26] have suggested a novel Superpixel-based Attention Graph Neural Network (SAGNN) for semantic segmentation of high spatial resolution aerial images. For each image, their network generates a K-Nearest Neighbor (KNN) graph, with each node representing a superpixel in the image and associated with a hidden representation vector. On this basis, the appearance feature extracted from the image by a unary Convolutional Neural Network (CNN) serves as the initialization of the hidden representation vector. Furthermore, each node can update its hidden representation based on the current state and incoming information from its neighbors using the attention mechanism and recursive functions. Each node’s final representation is used to predict the semantic class of each superpixel. Furthermore, superpixels not only save computational resources but also maintain object boundaries, resulting in more accurate predictions.

### 2.2 Problem statement

Deep learning approaches like CNN plays an essential role in the automatic discovery process in the field of Remote Sensing. But this deep learning approach required a huge number of data to train manually due to this the data annotation process gets lagged, and they are can’t able to use for the semantic segmentation process. The existing approaches utilized for semantic segmentation with deep learning approaches are showcased in Table 1. CAM-DFCN [19] automatically weights the feature maps of the channels to achieve effective feature selection. But, it may get lagged when a huge amount of data is utilized for segmentation and makes the system complex. ASPP [21] attained a huge number of abstract features by strengthening the network width and using the backbone network to perform semantic fusion in context to hold the number of spatial features. Yet, it faces a very high range of dissimilarity in the target ground because the images are attained from multiple regions. UVid-Net [24] provides highly accurate localization for class labels with the help of a feature refiner module and uses only a limited number of trainable parameters, and the computational complexity of the system is low. Still, it didn’t support the real-time system and also gets lagged when a camera is attained with a very high motion rate. CNN [18] utilized the statically collected training data to avoid fusion on particular mentioned classes. At the same time, it lost some important data at the time of acquiring the segmented feature map. OSM [22] consumes only a very low amount of time to train the given data. But, it didn’t provide a highly accurate outcome at the time of classification. MUNet [23] attained high-resolution segmented map outcomes from the road network. Yet, it achieved a very low accuracy rate with deep learning approaches. DSMF [20] is simple and it can be easily applied to all types of networks it can be trained easily and acquire effective features to attain better segmentation outcomes. But, it didn’t utilize any hand-designed components to enhance the performance of segmentation.

**Table 1:** Features and challenges in the conventional model for semantic segmentation.

Author [citation]	Methodology	Features	Challenges
Volpi and Tuia [18]	CNN	• It utilized the statically collected training data to avoid fusion on particular mentioned classes.	• It lost some important data at the time of acquiring the segmented feature map.
Luo et al. [19]	CAM-DFCN	• It automatically weights the feature maps of the channels to achieve effective feature selection.	• It may get lagged when a huge amount of data is utilized for segmentation and makes the system complex.
Cao et al. [20]	DSMF	• It is simple and it can be easily applied to all types of networks. • It can be trained easily and acquire effective features to attain better segmentation outcomes.	• It didn’t utilize any hand-designed components to enhance the performance of segmentation.
Liu et al. [21]	ASPP	• It attained a huge number of abstract features by strengthening the network width. • It uses a backbone network to perform semantic fusion in context to hold a number of spatial features.	• It faces a very high range of dissimilarity in the target ground because the images are attained from multiple regions.
Gupta et al. [22]	OSM	• It consumes only a very low amount of time to train the given data.	• It didn’t provide a highly accurate outcome at the time of classification.
Abdollahi et al. [23]	MUNet	• It attained high-resolution segmented map outcomes from the road network.	• It achieved a very low accuracy rate with deep learning approaches.
Girisha et al. [24]	UVid-Net	• It provides highly accurate localization for class labels with the help of a feature refiner module. • It uses only a limited number of trainable parameters and the computational complexity of the system is low.	• It didn’t support a real-time system. • It may get lagged when a camera is attained with a very high motion rate.

Thus, there is essential to develop a new advanced system for semantic segmentation of aerial images using deep learning approaches. Therefore, the AMC-Deeplabv3+ technique is designed for effectively segmenting the aerial images, where the parameters like epochs as well as the learning rate in the deeplabv3 model are optimized using the Improved Beluga Whale Optimization algorithm.

## 3. Dataset model and system architecture

### 3.1 Dataset model

The image data related to the semantic segmentation for the aerial images are regarded as the initial phase of the process. The relevant details about the required image data is obtained with the help of the following dataset links.

#### Dataset 1

This dataset is attained from “https://www.kaggle.com/humansintheloop/semantic-segmentation-of-aerial-imagery?select=Semantic+segmentation+dataset”: “Access Date: 2022-10-31”. It has been defined as the Semantic Segmentation of Aerial imagery. This dataset has acquired useful details about the aerial imagery of Dubai and it has been attained with the help of MBRSC satellites as well as annotated along with the pixel-wise semantic segmentation of six classes. It contains a total of 72 images that are grouped into 6 tiles.

#### Dataset 2

This dataset is attained from “http://jiangyeyuan.com/ASD/Aerial%20Image%20Segmentation%20Dataset.html”: “Access Date: 2022-10-31” [27]. It is named an aerial image segmentation dataset and it has been utilized in the research field for the Semantic Segmentation of Aerial Images. It has included 80 high-resolution images along with a spatial resolution that has range among 0.3 to 1.0. It also includes various scenarios such as power plants, warehouses, schools, and city as well as residential. The images are in 512-by-512 in size. Hence, the attained images data for SSAI are termed as $SS_{z}^{xz}$, and the total number of images gathered from the given dataset are indicated as *z* = 1,2,⋯;*Z*.

### 3.2 System architecture

In a huge amount of very high resolution (VHR), Remote Sensing images have been required on the daily basis with either space borne or airborne platforms that have been mainly dependent on the earth and mapping observations. Even though various research works have worked on the degree of automation for updating as well as on map generations has remained low. The manual representation of aerial images have been regarded as the classic issue of machine vision as well as Remote Sensing. Here, the semantically interpreted images such as thematic raster maps of the urban areas are highly essential for various applications like navigation, environmental monitoring, mapping and urban planning. The automatic segmentations into semantically well-determined classes are considered an active area for research for the last few years. This is particularly finite for urban areas as well as at high spatial resolutions. Here, the urban area has exhibited a huge variety of scheme in the reflectance. The situation has become even more difficult at the high spatial resolution. Urban land covers phases such as buildings or roads are regarded as the mixture of various materials and structures. Small objects like roof structures, individual cars, street furniture as well as things like traffic roads or signs markings have become visible. A benchmark technique for the segmentation issues has cast it as a supervised learning technique: has provided few labeled training data, and the statistical classifiers have learned to predict the conditional probabilities. Here, the input features are regarded as raw pixel intensities as well as various statistics or filter response has demonstrated the local image texture. In order to overcome the difficulties in the traditional model, this paper has implemented the new methodology for Semantic Segmentation of Aerial Images by using the newly recommended techniques, and its architectural depiction is shown in Fig 1. In this model, the aerial image segmentation process has been made by utilizing various phases.

**Fig 1:** Semantic segmentation of the aerial images architecture using the recommended models.

#### Encoder-decoder

These stages of the network are used on various computer vision-related tasks because of their effective performance. It has included the encoder step, which has the ability to capture high semantic information as well as consistently reduced the feature maps. On the other hand, the decoder step recovered the spatial details randomly. Therefore, sharper segmentation outcomes have been obtained through the Encoder-decoder phase in the DeepLabv3.

#### Encoder

This network has the ability to retrieve the relevant features by DCNN. Here, the output stride is regarded as region of the encoder module that depicts the spatial information about the output resolution before the global pooling or fully-connected layers. On regard to the semantic segmentation performance, the output stride has been attained as 16 to retrieve the denser features by employing the atrous convolutional as well as neglecting the striding on the two or one blocks. The encoder output is regarded as the last features map, which this features map has included 256 channels as well as richer semantic segmentations.

#### Decoder

This phase has failed to retain the entire object segmentation details. Therefore, there is a requirement for an effective decoder module, in which the bilinear upsampling of encoder features has been made through a factor of 4 and then integrated with equivalent low-level features through a network backbone that is similar to spatial resolution. At once, for performing the combination, the 3×3 convolution has been utilized for refining the features through bilinear upsampling. In the end, effective performance has been attained by using the output stride as 8 in the case of encoder phase.

#### Spatial pyramid pooling

It has been carried out on various grid scales that include the image-level pooling or has also been employed to different parallel atrous convolution along with various rates. This technique has been exploited on multi-scale details.

#### Depth-wise separable convolution

It has also been defined as the group convolutions that are the robust operation for minimizing the number of computational costs as well as parameters on capturing the slight betterment or similar working performance. This network has been factorized by the benchmark convolution into this network that is followed by 1×1 point-wise or convolution and thus, the computational complexity has been minimized. Specifically, the point-wise convolutional layer has been utilized for combining the depth-wise convolution; it has provided a spatial convolution network to the entire input channel. In depth-wise or spatial convolution, it has used atrous.

#### Atrous convolution

This phase is usually defined as the relevant tool for permitting the users for managing the resolution in the features, which is demonstrated through DCNN explicitly as well as adjusted the filters for producing the benchmark convolutional operation as well as managing multi-scale information.

In this model, they adopted a new Adaptive Multichannel deeplabv3+ model along with the aid of the developed IBWO algorithm, in which the hyper-parameters in the MC-Deeplabv3+ have been optimized by using the IBWO algorithm. The outcomes have shown that such a strategy has given better regularization over the series of strong baselines has reflected the ultra-modern techniques.

## 4. Implementing improved Beluga whale optimizer

### 4.1 Optimizing parameters and objective functions

In this phase, the deeplabv3 model has the ability to remove the noise from the images as well as it has been used to correct the contrast and density in the images. It has also been utilized to retrieve as well as store in the computer easily. But, it requires further development in error analysis and lighting variations. To tackle the difficulty, this technique has been optimized with the aid of the IBWO algorithm to further enhance the effectiveness of the Semantic Segmentation of Aerial images. The objective function used for the optimization is expressed in Eq (1).


$$ObFu=\underset{\left\{epch_{DLV3},LRT_{DLV3}\right\}}{\arg\;\min}(\frac{1}{Accr+dc})$$ (1)

Here, the objective function is denoted as *ObFu*, epochs in the Deplabv3 between [50–100] is termed *epch*_*DLV*3_ and the learning rate in Deplabv3 between [0.01–0.99] is defined as *LRT*_*DLV*3_ optimized in order to semantic segmentation outcomes for the aerial images with maximized dice coefficient and accuracy. Here, the dice coefficient is indicated *dc* and the accuracy is given as *Accr* and it is given in Eqs (2) and (3).


$$dc=\frac{2\times ra}{\left(ra+sg)+(ra+sg\right)}$$ (2)

$$acc=\frac{(rv+rn)}{\left(rv+rn+sm+sg)\right)}$$ (3)

Here the terms *sm*, *rn*, *sg* and *rv* refers to the “false positive, true negative, false negatives, and the true positive” accordingly.

### 4.2 Proposed IBWO for parameter optimization

Here, the new algorithm called IBWO for parameter optimization has been designed through BWO. The BWO algorithm is defined as the derivate-free optimization technique and it has the potential to balance both the exploitation and exploration stages to ensure global convergence. But it has faced difficulty in resolving discrete issues. To overcome the issues, the new IBWO is developed and the improvement is made on a random number.


$$h=alpha*(\frac{db}{A})$$ (4)

$$alpha=ObFu_{bestfitness}-ObFu_{worstfitness}$$ (5)

db=rand(bias) (6)

$$A=\frac{\left[mean(dis\tan ce(fitness-ObFu_{worstfitness}))\right)}{\left[mean(dis\tan ce(fitness-ObFu_{bestfitness}))\right)}$$ (7)

Here, the random number is denoted as *h* the best fitness is indicated as *ObFu*_*bestfitness*_, and *ObFu*_*worstfitness*_ is termed as worst fitness.

The BWO [28] algorithm has been developed by observing the foraging behaviour of whale that belongs to beluga whale (BW), which includes whale fall, swimming and preying. It is defined as a member of a whale living on the sea as well as it is familiar with pure white color adults and called a canary of the sea through generating various sounds. It has hearing ability and also has sharp vision as well as they propagate and hunt through its sound. Similar to all other algorithms, the BWO algorithm has also included three different phases. Here, the exploitation stage has the ability to manage the local search in the developed phase as well as the exploration stage has ensured the global searching capability in the developed space by using the random selection of BW. Some of the whales fall into the deep sea or may die at the time of migration which is defined as the whale fall. Even more, the probability function of the whale fall is regarded as in BWO that changed the location of the BW.

In the case of population dependent mechanism of the BWO, the beluga whale has considered the search agent, on each of the BW is determined as the candidate solution that is updated at optimizations. The matrix for the location of the searching agents is given in Eq (8)

$$G=[\begin{array}{cccc} g_{1,1} & g_{1,2} & \cdots & g_{1,a}\\ g_{2,1} & g_{2,2} & \cdots & g_{2,a}\\ \vdots & \vdots & \vdots & \vdots \\ g_{b,1} & g_{b,2} & \cdots & g_{b,a} \end{array})$$ (8)

Here, the dimension of the developed variables is termed as *a* and the population size of the beluga whale is indicated as *b*. For each beluga whale, the correspondent fitness value function is expressed as in Eq (9)

$$A_{g}=[\begin{array}{c} ai(g_{1,1},g_{1,2},\cdots ,g_{1,a})\\ ai(g_{2,1},g_{2,2},\cdots ,g_{2,a})\\ \vdots \\ ai(g_{b,1},g_{b,2},\cdots ,g_{b,a}) \end{array})$$ (9)

The BWO algorithms have converted from exploration into exploitation stage based on the balance factor *C*_*ai*_ that is expressed as in Eq (10).


$$C_{ai}=C_{0}(1-\frac{B}{2B_{\max}})$$ (10)

Here, the random changes among (0, 1) at all iteration is termed as *C*_0_ the current iteration is indicated as *B* well as the maximum iterative number is given as *B*_max_. The exploitation phase takes place when the value of *C*_*ai*_≤0.5 and the exploration phase is carried out when *C*_*ai*_>0.5.

#### Exploration phase

The exploration stage on the BWO has been demonstrated by regarded with the swimming mannerism of the beluga whale. On considering the documented behaviour of the beluga whale in human care, the beluga whale has performed the social-sexual mannerism under various postures like pair swims of two BW, which is closely together with the mirrored manner. Hence, the location of the searching agents is determined through the pair swim of BW as well as the location of the beluga whale is updated as given in Eq (11).


$$\left\{\begin{array}{cc} \begin{array}{l} G_{c,d}^{B+1}=\\ G_{c,e_{d}}^{B}+(G_{h,e_{c}}^{B}-G_{c,e_{d}}^{B})(1+h_{1})\sin(2\pi h_{2}), \end{array} & d=even\\ \begin{array}{l} G_{c,d}^{B+1}=\\ G_{c,e_{d}}^{B}+(G_{h,e_{c}}^{B}-G_{c,e_{d}}^{B})(1+h_{1})\cos(2\pi h_{2}) \end{array} & d=odd \end{array}\right)$$ (11)

Here, the random number among (0, 1) is denoted as *h*_1_*h*_2_, the new location for the *c*^*th*^ BW on the *d*^*th*^ dimension is given as $G_{c,d}^{B+1}$, the position of the *c*^*th*^ BW on the *e*_*c*_ dimension is given as $G_{c,e_{d}}^{B}$, the random number selected from *f* dimension is referred to as *e*_*c*_(*d* = 1,2,⋯,*f*), the current iteration is denoted as *B*, the current location for *c*^*th*^ and *h*^*th*^ BW termed as $G_{c,e_{d}}^{B}G_{h,e_{c}}^{B}$. The fins of the mirrored BW towards the surface are termed as sin(2*πh*_2_)cos(2*πh*_2_). On considering the dimension selected by even and odd numbers, the updated position has reflected the mirror or synchronous behaviours of BW on driving or swimming. Here, *h*_1_*andh*_2_ has been utilized to improve the random operators in the exploration phases.

#### Exploitation stage

Here, the exploitation stage of the BWO has been developed from the preying mannerism of the beluga whale. The beluga whale has cooperatively foraged as well as moved with respect to the location of the beluga whale. Hence, the BW preys through propagating the details of location for each other, regarding the best candidates as well as others. The strategy of the Levy flight has been implemented on the exploitation stage of BWO to improve the convergence. They can chase the prey along with the Levy flight strategy as well as the mathematical model that has been given in Eq (12).


$$G_{c}^{B+1}=h_{3}G_{bst}^{B}-h_{4}G_{c}^{B}+D_{1}•LF_{A}•(G_{h}^{B}-G_{c}^{B})$$ (12)

Here, the random number among (0, 1) is indicated as *h*_2_*h*_4_, the best location between BW termed as $G_{bst}^{B}$, the position of the new position of the *c*^*th*^ BW is indicated as $G_{c}^{B+1}$, the current position for the *c*^*th*^ beluga whale as well as the random beluga whale are given as $G_{h}^{B},G_{c}^{B}$. The current iteration is indicated as *B*. Here, the term $D_{1}=2h_{4}(1-\frac{B}{B_{\max}})$ refers to the random jump ability, which measures the intensity of Levy flight. The Levy flight function is termed as *LF*_*A*_ and it is indicated as in Eq (13).


$$LF_{A}=0.05\times \frac{i\times \omega }{{\left|j\right)}^{1/\xi }}$$ (13)

$$\omega =(\frac{\Gamma (1+\xi )\times \sin(\pi \xi /2)}{\Gamma ((1+\xi )/2)\times \xi \times 2^{(\xi -1)/2}})$$ (14)

Here, the default constant value equal to 1.5 is given *ξ* and the normally distributed random number is referred to as *i*,*j*

#### Whale fall

To assure the population size of the algorithm is constant, the location of BW, as well as the step size of the whale fall, has been utilized to demonstrate the updated position and it is expressed in Eq (15).


$$G_{c}^{B+1}=h_{5}G_{c}^{B}-h_{6}G_{h}^{B}+h_{7}G_{stp}$$ (15)

The step size of the whale fall is denoted as *G*_*stp*_, and the random number between (0, 1) is termed as = *h*_5_, *h*_,6_ *h*_7_.


$$G_{stp}=(U_{bo}-L_{bo})\exp(\frac{-D_{2}B}{B_{mx}})$$ (16)

Here, the upper and lower boundary of the variables is indicated *U*_*bo*_,*L*_*bo*_ accordingly. The step factor is given as *D*_2_.

In this technique, the probability of whale fall *Z*_*ai*_ has been computed as a linear function as given in Eq (17).


$$Z_{ai}=\frac{0.1-0.05B}{B_{mx}}$$ (17)

The whale fall probability in the last iteration is 0.05 that is reduced from the initial iteration to 0.1 and the pseudo-code for the segmentation of aerial images is given in Algorithm 1.

**Algorithm 1: IBWO**

Initialize the population size and maximum iteration

While *B*≤*B*_*mx*_

 Compute the value of *h* using Eq (4)

 Attain *Z*_*ai*_ and *C*_*ai*_ using Eqs (17) and (10)

  If *C*_*ai*_(*c*)>0.5

   Update new position in the exploration phase using Eq (11)

  Else

   Update new position in the exploitation phase using Eq (12)

  End if

   If *C*_*ai*_(*c*)≤*Z*_*ai*_

    Update new position in whale fall using Eq (15)

   End if

End while

End

Output best solution

The flowchart for the IBWO algorithm for the Semantic Segmentation of Aerial Images is depicted in Fig 2.

**Fig 2:** Flowchart for the IBWO algorithm for segmentation of aerial images.

## 5. A novel adaptive multichannel Deeplabv3+

### 5.1 DeepLabv3+ model

This technique has been similar to that of U-Net and has been utilized as the convolutional model that has an encoder-decoder structure. These stages of the network are used on various computer vision-related tasks because of their effective performance. It has included the encoder step, which has the ability to capture high semantic information as well as consistently reduced the feature maps. On the other hand, the decoder step recovered the spatial details randomly. Therefore, sharper segmentation outcomes have been obtained through the Encoder-decoder phase in the DeepLabv3. Dilated convolution is regarded as the kind of convolution employed to input along with the defined gaps. The dilation rate is defined as skipping pixels. Deeplabv3+ has utilized the Xception module for feature extractors as well as its output is considered a feature map, which is 1/16 the size of the traditional spectrogram. The term *l* = 1 denotes normal convolution. The encoder block has been considered as the convolutional neural network, which has retrieved the high-level features. In the initial phase, the encoder features have been bilinearly upsampled by the factor of 4 as well as it has been then concatenated along with the corresponding low-level features through the network backbone, which has a spatial resolution.

After the concatenation, the 3 × 3 convolutions have been employed in order to regain the features that have been followed by other bilinear upsampling by the factor value of 4. The decoder blocks then attained the mask spectrogram of the similar size as an input spectrogram. On neglecting the connection on the third layer, a high-resolution function map has easily been transformed. When the magnitude spectrogram of the target audio is defined as *L* well as the input spectrogram of the mixed signal is indicated *M* then the loss function values have been utilized to train the model is the MSE of the difference among the masked input spectrogram as well as the target spectrogram is represented in Eq (18).


$$N(L,M)={\left\|v(L)•L_{mg}-M\right)}_{2}$$ (18)

Here, the element-wise product indicated as • well as the output of the network is given as *v*(*L*), and the magnitude spectrograms of the reference microphone are termed as *L*_*mg*_. The DeepLabv3+ model for semantic segmentation is shown in Fig 3.

**Fig 3:** DeepLabv3+ model for semantic segmentation.

### 5.2 Multichannel Deeplabv3+ model

The multi-channel structure has been demonstrated as it has the ability to learn the local body-parts features as well as the global full-body features jointly and then, the fusion of these two features has been made at the final phase to improve the accuracy of the model. It has also been utilized for image classifications. Every channel has the ability to process the small images into various parts of the large images as well as extract the features. The channel is composed of certain layers and it has been integrated into a common fully connected layer. On top of the entire technique, one output layer has provided the required outcomes. It has also included the training phase, after the training phase, the classifiers have classified the images. These techniques have the ability to perform well even in a resource-limited computing environment and the multichannel Deeplabv3+ model for segmentation is given in Fig 4.

**Fig 4:** Diagrammatic depiction of multichannel Deeplabv3+ model for segmentation.

### 5.3 Adaptive Multichannel Deeplabv3+ model

In this phase, the AMC-DeepLabV3+ has been implemented with the help of the IBWO algorithm in order to design the semantic segmentation of the model of the aerial image. The DeepLabV3+ model has the potential to enhance the density of the features as well as extend the receptive fields. Here, the residual structure can also resolve the degradation issues caused by the deep network. But, it has faced issues, in which the bilinear upsampling techniques are not good enough to retain more details. The Deeplabv3 has the ability to assign a label to each pixel in the image. But, it has failed to scale as well as larger DCNN due to limited GPU memory. In order to tackle the issues in the model, the AMC-DeepLabV3+ has been designed, where the parameters like epochs and the learning rate are optimized with the help of the IBWO algorithm. Here, the input $SS_{z}^{xz}$ is given as the input, as well as the output, is attained as semantic segmented aerial images with higher or maximized values of accuracy and dice-coefficient that enhance the performance of the recommended model and the AMC-DeepLabV3+ model is given in Fig 5.

**Fig 5:** Diagrammatic representation of the AMC-DeepLabV3+ model.

## 6. Results and discussions

To enhance the accuracy and Dice coefficient by concerning a multi-objective function, proposing an improved Beluga Whale optimizer derived Adaptive Multi-channel Deeplabv3+ for semantic segmentation of Aerial images by the involvement of both encoder-decoder structure and spatial pyramid pooling module. The findings of the designed method provides improved accuracy and dice coefficient with lower computation time in the segmentation of small buildings, roads and trees, while also having a more realistic shape. When it comes to the segmentation of large buildings, the target boundary is more accurate, with no obvious voids, and the segmentation effect is noticeably enhanced. It is utilized for the critical applications like robotic navigation, scene understanding, autonomous driving, and localization.

### 6.1 Experimental setup

The proposed Semantic segmentation of Aerial Images has been implemented in Python, and the experimental investigation was done using the Ubuntu operating system and a 16 GB RAM NVIDIA Tesla P100 GPU. The installed software consists of CUDA 11.0, Tensor flow 2.1.0, and Keras deep learning framework (version 2.3.0). Here, the performance of the Semantic segmentation of Aerial Images has been assimilated over the conventional models in terms of metrics like Accuracy and Dice Coefficient. The algorithms such as Butterfly Optimization Algorithm (BOA) [29], Coyote Optimization Algorithm (COA) [30], Glow-worm Swarm Optimization (GSO) [31], and classifiers like UNet [32], Deeplabv3 [33], MC-Deeplabv3 [34] and G-RDA-Deeplabv3[35] has been utilized for assimilation over AMC-DeepLabV3+ model. The maximum Iteration was 10; the chromosome length was 2 as well as the number of Populations was 10. Initially, the data are gathered from the dataset in section 3.1. Then, the given data are taken as 100%, from this, 70% of the data are used for training and 30% of the data are used for testing the proposed model to show the efficiency of the model even tested with the minimum amount of data.

### 6.2 Semantic segmentation outcomes

The Semantic Segmentation outcomes shows the segmentation effects of the UNet, DeepLabV3 and the proposed Adaptive Multi-channel DeepLabv3+ model. When compared to UNet, DeepLabV3 and the model suggested in this paper shows higher accuracy in the segmentation of small buildings, roads and trees, while also having a more realistic shape. When it comes to the segmentation of large buildings, the target boundary is more accurate, with no obvious voids, and the segmentation effect is noticeably enhanced.

### 6.3 Statistical analysis on various algorithms

Here, Figs 6 and 7 and Tables 2 and 3 has represented the statistical analysis for the semantic segmentation on various algorithms for both dataset 1 and 2 respectively. The value of IBWO-AMC-DeepLabV3+ has shown betterment over other models. The value of accuracy of IBWO-AMC-DeepLabV3+ is 9.6%, 8.4%, 6.0%, and 4.9% higher than BOA-AMC-DeepLabV3+, COA-AMC-DeepLabV3+, GSO-AMC-DeepLabV3+, and BWO-AMC-DeepLabV3+ at best for dataset 1. Consequently, for dataset 2, 13.5%, 12.2%, 9.7% and 9.7% higher than BOA-AMC-DeepLabV3+, COA-AMC-DeepLabV3+, GSO-AMC-DeepLabV3+, and BWO-AMC-DeepLabV3+ at best. Similarly, the value of Dice coefficient of IBWO-AMC-DeepLabV3+ is 10.2%, 8.8%, 5.2%, and 5.1% higher than BOA-AMC-DeepLabV3+, COA-AMC-DeepLabV3+, GSO-AMC-DeepLabV3+, and BWO-AMC-DeepLabV3+ at best for dataset 1. Consequently, for dataset 2, 11.9%, 10.4%, 8.1% and 8.3% higher than BOA-AMC-DeepLabV3+, COA-AMC-DeepLabV3+, GSO-AMC-DeepLabV3+, and BWO-AMC-DeepLabV3+ at best. Hence, the value of IBWO-AMC-DeepLabV3+ has shown maximum values for the Semantic Segmentation of Aerial Images.

**Fig 6:** Performance analysis for the semantic segmentation of aerial images using algorithms for dataset 1 regarding (a) accuracy and (b) Dice coefficient.

**Fig 7:** Performance analyses for the semantic segmentation of aerial images using algorithms for dataset 2 regarding (a) accuracy and (b) Dice coefficient.

**Table 2:** Statistical analysis for semantic segmentation on various algorithms for dataset 1.

Performance Metrics	Terms	BOA-AMC DeepLabV3+ [29]	COA-AMC DeepLabV3+ [30]	GSO-AMC DeepLabV3+ [31]	BWO-AMC DeepLabV3+ [28]	IBWO-AMC Deeplabv3+
**Accuracy**	Best	0.9	0.91	0.93	0.94	0.98645
	Worst	0.82	0.83	0.84	0.84	0.97689
	Mean	0.858	0.872	0.878	0.88	0.97423
	Median	0.855	0.87	0.87	0.875	0.98352
	Standard deviation	0.027857	0.030919	0.032496	0.034351	0.00337
**Dice Coefficient**	Best	0.895833	0.907216	0.927835	0.938776	0.987368
	Worst	0.8125	0.824742	0.833333	0.833333	0.986735
	Mean	0.852384	0.867245	0.873944	0.876427	0.987051
	Median	0.849764	0.864583	0.865979	0.87049	0.987412
	Standard deviation	0.029038	0.031907	0.033594	0.035582	0.0034183

**Table 3:** Statistical analysis for semantic segmentation on various algorithms for dataset 2.

Performance Metrics	Terms	BOA-AMC DeepLabV3+ [29]	COA-AMC DeepLabV3+ [30]	GSO-AMC DeepLabV3+ [31]	BWO-AMC DeepLabV3+ [28]	IBWO-AMC Deeplabv3+
**Accuracy**	Best	0.87	0.88	0.9	0.9	0.98721
	Worst	0.79	0.8	0.82	0.83	0.97589
	Mean	0.827	0.841	0.864	0.875	0.97323
	Median	0.825	0.84	0.86	0.88	0.97352
	Standard deviation	0.029343	0.025865	0.028355	0.023345	0.00337
**Dice Coefficient**	Best	0.882883	0.894737	0.913793	0.912281	0.98854
	Worst	0.814159	0.824561	0.842105	0.849558	0.987735
	Mean	0.846871	0.859536	0.880642	0.8904	0.986051
	Median	0.847216	0.858407	0.877107	0.894652	0.986412
	Standard deviation	0.025485	0.023503	0.025055	0.020751	0.003418

### 6.4 Statistical analysis on various classifiers

Here, the statistical analyses for the semantic segmentation on various classifiers are represented in Figs 8 and 9 and Tables 4 and 5 for both dataset respectively. The value of IBWO-AMC-DeepLabV3+ has shown better outcomes over other conventional classifiers. The value of the accuracy of IBWO-AMC-DeepLabV3+ is 3%, 2.1%, 1.4%, and 1% higher than UNet, Deeplabv3, MC-Deeplabv3 and G-RDA-Deeplabv3 at best for dataset 1. Consequently, for dataset 2, 3.1%, 2.2%, 1.3% and 1.1% higher than UNet, Deeplabv3, MC-Deeplabv3 and G-RDA-Deeplabv3 at best. Similarly, The value of the dice coefficient of IBWO-AMC-DeepLabV3+ is 2.9%, 2.1%, 0.8%, and 0.5% higher than UNet, Deeplabv3, MC-Deeplabv3 and G-RDA-Deeplabv3 at best for dataset 1. Consequently, for dataset 2, 3%, 2.2%, 0.9% and 0.7% higher than UNet, Deeplabv3, MC-Deeplabv3 and G-RDA-Deeplabv3 at best Hence, the value of IBWO-AMC-DeepLabV3+ has shown maximum values for the Semantic Segmentation of Aerial Images.

**Fig 8:** Performance analysis for the semantic segmentation of aerial images using classifiers for dataset 1 regarding (a) accuracy and (b) Dice coefficient.

**Fig 9:** Performance analyses for the semantic segmentation of aerial images using classifiers for dataset 2 regarding (a) accuracy and (b) Dice coefficient.

**Table 4:** Statistical analysis for semantic segmentation on various classifiers for dataset 1.

Performance Metrics	Terms	UNet [32]	Deeplabv3 [33]	MC-Deeplabv3 [34]	G-RDA-DeepLabv3 [35]	IBWO-AMC-Deeplabv3+
**Accuracy**	Best	0.956894	0.965454	0.97275	0.976196	0.98645
	Worst	0.946854	0.959167	0.964836	0.974747	0.97689
	Mean	0.952299	0.962328	0.973728	0.975533	0.97423
	Median	0.952667	0.962296	0.974091	0.975548	0.98352
	Standard deviation	0.002715	0.001782	0.004336	0.00028	0.00337
**Dice Coefficient**	Best	0.958715	0.966786	0.979298	0.98176	0.987368
	Worst	0.949351	0.960676	0.971541	0.980229	0.986735
	Mean	0.954469	0.963678	0.975419	0.981042	0.987051
	Median	0.954534	0.963653	0.975513	0.981045	0.987412
	Standard deviation	0.002483	0.001694	0.056433	0.000266	0.0034183

**Table 5:** Statistical Analysis for semantic segmentation on various classifiers for dataset 2.

Performance Metric	TERMS	UNet [32]	Deeplabv3 [33]	MC-Deeplabv3 [34]	G-RDA-Deeplabv3 [35]	IBWO-AMC-Deeplabv3+
**Accuracy**	Best	0.956863	0.965378	0.974521	0.976166	0.98721
	Worst	0.946381	0.959137	0.962638	0.974686	0.97589
	Mean	0.951606	0.962381	0.968579	0.975563	0.97323
	Median	0.951508	0.962608	0.968741	0.975586	0.97352
	Standard deviation	0.002949	0.001854	0.004336	0.000304	0.00337
**Dice Coefficient**	Best	0.958843	0.966684	0.979312	0.981698	0.98854
	Worst	0.948863	0.960746	0.971412	0.980226	0.987735
	Mean	0.953823	0.96376	0.975362	0.981078	0.986051
	Median	0.953689	0.963998	0.975135	0.981114	0.986412
	Standard deviation	0.002694	0.001755	0.056433	0.000293	0.003418

### 6.5 Overall analysis on various state of art approaches

Here, the Analysis for the semantic segmentation of aerial images over the existing state of art techniques from past literature has been evaluated and it is tabulated in Table 6 for dataset 1 and 2. The proposed IBWO-AMC-Deeplabv3+ has 12.8%,12.4% and 13.6% higher in terms of accuracy in dataset 1 over CNN, MUnet and DFCNN models. Consequently, for dataset 2, 3.2%,8.1% and 4% higher in terms of accuracy over CNN, MUNet and DFCNN models. Hence it has proven that the suggested IBWO-AMC-Deeplabv3+ has outperformed and superior over other models. Similarly, in terms of dice coefficient for dataset 1, the proposed IBWO-AMC-Deeplabv3+ has 12.7%, 11.9% and 13.7% higher over CNN, MUnet and DFCNN models. Consequently, for dataset 2, the dice coefficient of IBWO-AMC-Deeplabv3+ has 9.4%, 14.7% and 10.4% higher over CNN, MUnet and DFCNN models. Fig 10 represents the overall Analysis for Semantic Segmentation on Various State of Art from Past literature for Dataset 1 and 2.

**Fig 10:** Overall analysis for semantic segmentation on various state of art from past literature for dataset 1 and 2.

**Table 6:** Overall analysis for semantic segmentation on various state of art from past literature for dataset 1 and 2.

Datasets	Performance metrics	CNN [18]	DFCNN [19]	MUnet [23]	IBWO-AMC-Deeplabv3+
Dataset 1	Accuracy	0.874146	0.868195	0.877579	0.98645
	Dice Coefficient	0.876048	0.868279	0.881787	0.987368
Dataset 2	Accuracy	0.901077	0.893463	0.859619	0.98721
	Dice Coefficient	0.9027	0.894735	0.86122	0.98854

## 6.6 Computational complexity

Here, the Computational time for semantic segmentation of Aerial images for various Algorithms, Classifiers and state of the art techniques were evaluated and tabulated in Table 7. The proposed Adaptive Multi-channel DeepLabv3+ (AMC-DeepLabv3+) model has 9.25%, 1.9%, 8.44% lesser in terms of computational time over the Algorithms BOA-AMC-DeepLabv3+, COA- AMC-DeepLabv3+, GSO- AMC-DeepLabv3+ and 0.75% higher over BWO- AMC-DeepLabv3+. Similarly comparing over the state of the art techniques like CNN, MUnet and DFCNN, the AMC-DeepLabv3+ has 10.06%, 3.28% and 9.74% lesser computation time. And also, the AMC-DeepLabv3+ has 6.69%, 15.86%, 2.45% and 5.21% lesser over the various classifiers like UNet, DeepLabV3, MC-DeepLabV3 and G-RDA-DeepLabv3. Therefore, the proposed model achieves less Computational time for the semantic segmentation of aerial images over various Algorithms, Classifiers and the state of the art techniques.

**Table 7:** Computational complexity over various algorithms and classifier models.

Algorithms / Classifiers	Models	Execution time in Seconds
**Algorithms**	BOA-AMC-DeepLabv3+ [29]	124.5365
	COA- AMC-DeepLabv3+ [30]	115.2364
	GSO- AMC-DeepLabv3+ [31]	123.4359
	BWO- AMC-DeepLabv3+ [28]	112.1546
**Classifiers**	CNN [18]	125.6548
	Munet [23]	116.8564
	DFCNN [19]	125.2145
	UNet [32]	121.1228
	DeepLabV3 [33]	134.3211
	MC-DeepLabV3 [34]	115.8564
	G-RDA-DeepLabv3 [35]	119.2324
	**IBWO-AMC-Deeplabv3+**	**113.0123**

### 6.7 Ablation analysis

Abalation Experiments were conducted on both semantic segmentation of aerial imagery and Aerial image segmentation data sets. In comparison to DeepLabV3 and MC-DeepLabv3, the AMC-DeepLabv3+ displays more accuracy in the segmentation of minor structures, roads, and trees while also having a more realistic form. The target border for the segmentation of huge structures is more precise, with no noticeable voids, and the segmentation impact is substantially improved. Ablation Analysis of AMC-DeepLabv3+ on dataset 1 and 2 are depicted in Tables 8 and 9 respectively.

**Table 8:** Ablation analysis of AMC-DeepLabv3+ on dataset 1.

Model	Accuracy (%)	Dice Coefficient (%)
DeepLabv3	96.5454	96.6686
MC-DeepLabv3	97.4575	97.9398
IBWO-AMC-DeepLabv3+	**98.7245**	**98.8568**

The value of IBWO-AMC-DeepLabV3+ has shown better outcomes over other conven-tional classifiers. The value of the accuracy of IBWO-AMC-DeepLabV3+ is 2.1% and 1.4% higher than Deeplabv3, MC-Deeplabv3 at best for dataset 1. Similarly The value of the dice coefficient of IBWO-AMC-DeepLabV3+ is 2.1% and 0.8% higher than Deeplabv3 and MC-Deeplabv3 at best for dataset 1.

**Table 9:** Ablation analysis of AMC-DeepLabv3+ on dataset 2.

Model	Accuracy (%)	Dice Coefficient (%)
DeepLabv3	96.5378	96.6684
MC-DeepLabv3	97.4521	97.9312
IBWO-AMC-DeepLabv3+	**98.7210**	**98.8540**

The value of IBWO-AMC-DeepLabV3+ has shown better outcomes over other conven-tional classifiers. The value of the accuracy of IBWO-AMC-DeepLabV3+ is 2.2% and 1.3% higher than Deeplabv3, MC-Deeplabv3 at best for dataset 2. Similarly The value of the dice coefficient of IBWO-AMC-DeepLabV3+ is 2.2% and 0.9% higher than Deeplabv3 and MC-Deeplabv3 at best for dataset 2.

## 7. Conclusion

In this work, an enhanced multi-objective derived adaptive multichannel DeepLabv3+ using an improved Beluga Whale optimization algorithm is implemented for the semantic segmentation of aerial images. The proposed Adaptive Multichannel DeepLabv3+ employs an encoder-decoder structure in which DeepLabv3 is used to encode the rich contextual information and a simple yet effective decoder module is used to recover the object boundaries. Depending on the available computation capabilities, the atrous convolution could also be used to extract encoder characteristics at various resolutions. We also investigate the Xception model as a backbone network with atrous separable convolution to make the proposed model faster and stronger. This model has effectively segmented the aerial images semantically and the hyperparameters in the AMC-DeepLabV3+ model such as epochs and learning rate were optimized by the Improved Beluga Whale Optimization algorithm.

The proposed AMC-DeepLabv3+ is evaluated on two publicly available datasets, semantic segmentation of aerial imagery and Aerial image segmentation. The semantic segmented aerial images have achieved maximized accuracy and dice coefficient. With the dataset 1, the proposed AMC-Deeplabv3+ achieved the best results as improved accuracy of 98.64%, Dice coefficient of 98.73%. Likewise with dataset 2, achieved the best results as improved accuracy of 98.74%, Dice coefficient of 98.83%. The performance the proposed IBWO-AMC-Deeplabv3+ has 12.8%,12.4% and 13.6% higher in terms of accuracy in dataset 1 over CNN, MUnet and DFCNN models. Consequently, for dataset 2, 3.2%, 8.1% and 4% higher in terms of accuracy over CNN, MUNet and DFCNN models. In terms of Dice-coefficient, the proposed model has 12.70%, 11.97%, and 13.71% higher in dataset 1 over CNN, MUnet and DFCNN models. Consequently, for dataset 2, 9.4%, 14.76% and 10.46% higher over CNN, MUnet and DFCNN models. Therefore, the evolutional outcomes of the proposed AMC-DeepLabv3+ model shows significantly better than the state-of-the-art models on both datasets.

Hence, it further has assured the effectiveness of the recommended semantic segmentation of the aerial images. This model suffers from a lack of processing the large-scale datasets in this semantic segmentation of aerial image that are harder to design real-time segmentation. It is significant to detect the trade-off value among accuracy and run-time. Segmentation process generally requires more memory space for execution in terms of both training and interference, enhancing the memory space, which will be considered in future for promoting the performance.

## Abbreviation Description

CNN: Convolutional Neural Networks
DCNN: Deep Convolutional Neural Network
IBWO: Improved Beluga whale optimization
FCN: Fully Convolutional Neural Network
IRRG: Infrared, Red, and Green
DRN: Deep Residual Networks
DFCN: Deep Fully Convolutional Network
CAM-DFCN: Channel Attention Mechanism-Deep Fully Convolutional Neural Network
ASPP: Atrous Spatial Pyramid Pooling
UAV: Unmanned Aerial Vehicle
OSM: Open Street Map
GAN: Generative Adversarial Network
DSM: Digital Surface Models
DSMF: Digital Surface Models Fusion
FoV: Field-of-View
VHR: Very High Resolution
BWO: Beluga Whale Optimization
GSO: Glow-worm Swarm Optimization
BOA: Butterfly Optimization Algorithm
COA: Coyote Optimization Algorithm
